The article "Heat Shock Protein 90 (HSP90) Inhibitors as Anticancer Medicines: A Review on the Computer-Aided Drug Discovery Approaches over the Past Five Years" was published in 2022. Journal: Comput Math Methods Med.

# Heat Shock Protein 90 (HSP90) Inhibitors as Anticancer Medicines: A Review on the Computer-Aided Drug Discovery Approaches over the Past Five Years

**DOI:** 10.1155/2022/2147763

**Published:** 2022-05-31

**Authors:** Ayanda M. Magwenyane, Samuel C. Ugbaja, Daniel G. Amoako, Anou M. Somboro, Rene B. Khan, Hezekiel M. Kumalo

**Affiliations:** ^1^Drug Research and Innovation Unit, Discipline of Medical Biochemistry, School of Laboratory Medicine and Medical Science, University of KwaZulu-Natal, Durban 4000, South Africa; ^2^Biomedical Resource Unit, College of Health Sciences, University of KwaZulu-Natal, Durban 4000, South Africa

## Abstract

Cancer is a disease caused by the uncontrolled, abnormal growth of cells in different anatomic sites. In 2018, it was predicted that the worldwide cancer burden would rise to 18.1 million new cases and 9.6 million deaths. Anticancer compounds, often known as chemotherapeutic medicines, have gained much interest in recent cancer research. These medicines work through various biological processes in targeting cells at various stages of the cell's life cycle. One of the most significant roadblocks to developing anticancer drugs is that traditional chemotherapy affects normal cells and cancer cells, resulting in substantial side effects. Recently, advancements in new drug development methodologies and the prediction of the targeted interatomic and intermolecular ligand interaction sites have been beneficial. This has prompted further research into developing and discovering novel chemical species as preferred therapeutic compounds against specific cancer types. Identifying new drug molecules with high selectivity and specificity for cancer is a prerequisite in the treatment and management of the disease. The overexpression of HSP90 occurs in patients with cancer, and the HSP90 triggers unstable harmful kinase functions, which enhance carcinogenesis. Therefore, the development of potent HSP90 inhibitors with high selectivity and specificity becomes very imperative. The activities of HSP90 as chaperones and cochaperones are complex due to the conformational dynamism, and this could be one of the reasons why no HSP90 drugs have made it beyond the clinical trials. Nevertheless, HSP90 modulations appear to be preferred due to the competitive inhibition of the targeted N-terminal adenosine triphosphate pocket. This study, therefore, presents an overview of the various computational models implored in the development of HSP90 inhibitors as anticancer medicines. We hereby suggest an extensive investigation of advanced computational modelling of the three different domains of HSP90 for potent, effective inhibitor design with minimal off-target effects.

The article "Heat Shock Protein 90 (HSP90) Inhibitors as Anticancer Medicines: A Review on the Computer-Aided Drug Discovery Approaches over the Past Five Years" was published in 2022. Journal: Comput Math Methods Med.

## 1. Introduction

Cancer is a term used to describe a collection of diseases defined by the uncontrolled development, growth, and spread of aberrant cells outside their normal bounds. According to World Health Organization (WHO) data, cancer is the second biggest cause of mortality worldwide, accounting for 9.6 million fatalities in 2018, or one in every six deaths [1–3]. The repeated upsurge of specific cancers is caused by several factors, including population expansion, ageing, and the altering forms of cancer determinants which could be socially or economically related [4]. Aside from the earlier mentioned concerns, lifestyle-related and physical behaviours such as nutrition, alcohol usage, and physiological behaviours have all been linked to cancer risk and burden [1, 5]. Cancer can also be described as a group of diseases caused by cells' uncontrolled, abnormal growth in different anatomic sites [6]. New cells arise while old cells die in a natural, harmless cycle of dividing cells. Cancer disturbs cell division, causing old cells to persist and new cells to form prematurely, resulting in tumours visible as aberrant cell proliferation that causes swelling. It is important to note that some malignancies, such as leukaemia, do not form tumours and are identified in the bloodstream [6]. There are two sorts of tumours: benign and malignant. Benign tumours are noncancerous but can grow. However, such tumours do not grow and are noninvasive. In addition, benign tumours do not develop back when successfully removed through surgery. For example, the outcome may be fatal if a benign tumour is found pressing on the brain or other vital organs [7]. Cancerous growths are referred to as malignant tumours and can be aggressively and uncontrollably replicated [8]. Another characteristic feature of malignant tumours is their ability to metastasise, a process of invading other body parts [9]. Cancer progress depends on external as well as internal factors, including those of the environment. The external considerations include cigarette/tobacco products, radiation, and infectious species.

On the other hand, genetic mutations, hormonal abnormalities of the immune system, and mutated metabolism are some of the internal aetiologies of cancer [10]. Tobacco use kills seven million people every year globally, with two-thirds of users expected to die from the disease. Smoking accounts for 22 percent of global cancer fatalities [11]. A weekly dose of a single wine bottle is predicted to have an increased absolute lifetime cancer risk of 1.0 percent and 1.4 percent for nonsmoking males and females, respectively [11]. The absolute average cancer risk increase for one bottle of wine per week is equivalent to five (men) or ten cigarettes per week (women) [11]. More than 20 percent of deaths from cancer in the developed world arise from infections that include hepatitis B and C viruses as well as human papillomavirus [12]. Hereditary abnormalities are thought to be the cause of 5–10% of cancers. In 2018, it was predicted that the worldwide cancer burden would rise to 18.1 million new cases and 9.6 million deaths. In the worldwide setting, 1 in 5 men and 1 in 6 women develop cancer over their lifetime, with 1 in 8 men and 1 in 11 women succumbing to the disease. The 5-year prevalence, or the number of persons living within five years following a cancer diagnosis, is predicted to be 43.8 million people worldwide [13]. Most common cancers remain undetected for months or even years due to slow accumulation of their mutations. DNA mutations usually occur at a rate of 1 in every 20 million genes per cell division [6].

The article "Heat Shock Protein 90 (HSP90) Inhibitors as Anticancer Medicines: A Review on the Computer-Aided Drug Discovery Approaches over the Past Five Years" was published in 2022. Journal: Comput Math Methods Med.

Sequel to the stress resulting from the ongoing research, researchers and pharmaceutical industries are under significant pressure to design and develop highly selective and efficient drugs for the treatment and management of various deadly cancers [1].

Anticancer compounds, often known as chemotherapeutic medicines, have gained much interest in recent cancer research [14]. These medicines work through various biological processes in targeting cells at multiple stages of the cell's life cycle. Recently, advancements in new drug development methodologies and the prediction of the targeted interatomic and intermolecular ligand interaction sites have been beneficial. This has prompted further research into developing and discovering novel chemical species as preferred therapeutic compounds against specific cancer kinds [15]. One of the most significant roadblocks in developing anticancer drugs is that traditional chemotherapy affects normal cells and cancer cells, resulting in substantial side effects [1]. Identifying new drug molecules with high selectivity and specificity for cancer is, therefore, a prerequisite in treating and managing the disease [1, 15]. There is a literature gap in terms of recent experimental and, in particular, computational data on the design and development of new HSP90 inhibitors. As a result, this review offers an insightful update on the various computational models implored in the development of HSP90 inhibitors as anticancer medicines over the past five years (2016 to 2021).

## 2. Overview of Some Cancer Therapeutic Targets for Drug Discovery

For many decades, care for patients with cancer was limited to only a few options. This included surgery, radiation therapy for minor solid tumours, and chemotherapy for blood cancers and solid metastatic tumours [16]. Human protein tyrosine kinases (PTKs) have a significant contribution to human cancer development and have surfaced as potential targets for cancer prevention [17, 18]. The discovery of small-molecule species with high selectivity and specificity to inhibit targeted proteins with cancer cells appears to be the brilliant strategy in cancer therapy. The epidermal growth factor receptor (EGFR) overexpression has been detected in most cancers. Therefore, targeting EGFR (proteins that attach to epidermal growth factors) has been one of the effective cancer therapies. Rapid cell division occurs when there is an overexpression of EGFR [19]. These EGFR proteins play a significant role in the signal's transmission network responsible for the survival and division of cells. Over the years, discovering small-molecule inhibitors of EGFR tyrosine kinase has attracted more significant resources from the pharmaceutical industry [20]. Overexpression of EGFR is linked to a poor clinical outcome in a variety of cancers, including cancers of the head and neck, larynx, oesophagus, stomach, pancreas, colon, renal cell, bladder, breast, ovaries, cervix, prostate, non-small-cell lung (NSCL) cancer, papillary thyroid cancers, melanoma, and gliomas [21]. Recently, numerous EGFR tyrosine kinase inhibitors (TKIs) have been identified, including canertinib, erlotinib, and gefitinib. Nevertheless, there are still current research studies towards discovering more potent and effective EGFR inhibitors due to some observed resistance to the available inhibitors [22].

The article "Heat Shock Protein 90 (HSP90) Inhibitors as Anticancer Medicines: A Review on the Computer-Aided Drug Discovery Approaches over the Past Five Years" was published in 2022. Journal: Comput Math Methods Med.

Researchers have also targeted cyclin-dependent protein kinases (CDKs) in the treatment of cancer. CDKs are essential proteins responsible for regulating the expression of most transmission mechanisms via the cell cycles [23]. In addition, the CDKs contribute immensely to other cell cycle mechanisms such as functions of the neurons, metabolic activities, and gene transcriptions [23]. Cyclin-dependent kinases (CDKs) are serine/threonine kinases responsible for protein phosphorylation on serine and threonine residues [24, 25]. According to studies, the overactivity of CDKs or inoperative CDK-inhibiting proteins is observed in some malignancies, thereby serving as promising targets for anticancer drugs [26]. Therefore, the development and design of drugs targeting CDK overexpression became imperative. Some CDK inhibitors, such as seliciclib, a cyclin-dependent kinase (CDK) inhibitor tested as an anticancer treatment, are already in phase II clinical trials [27, 28].

Another cancer treatment target is poly(ADP-ribose) polymerase (PARP), a common nuclear enzyme that is a marker of deoxyribonucleic acid (DNA) damage. The DNA repair enzyme poly(ADP-ribose) polymerase (PARP) shows significant and abundant expression in the nucleus of mammals. Researchers have been so interested in PARP due to its structural and fascinating inhibition properties [29]. The Food and Drug Administration (FDA) has approved several PARP inhibitors, targeting several cancer types [30]. These PARP inhibitors also operate as radiosensitisers by delaying single-strand break reparation. These inhibitors subsequently promote double-strand break production, a hypothesis that has been used in many preclinical combinatory models of PARP inhibitor and ionising radiation therapy [30]. In addition, this enzyme aids DNA repair by facilitating ADP-ribosylation of DNA, histones, and several DNA repair enzymes [31].

The article "Heat Shock Protein 90 (HSP90) Inhibitors as Anticancer Medicines: A Review on the Computer-Aided Drug Discovery Approaches over the Past Five Years" was published in 2022. Journal: Comput Math Methods Med.

For several illnesses, including cancer, PARPs have been the target of intensive structure-based drug design efforts. Some common examples of PARP targeted inhibitors include iniparib in the phase I trial, while BMN-673 and olaparib are in phase II clinical trials [32]. However, while traditional cancer therapies such as radiation and chemotherapy are effective, heat shock protein 90 (HSP90) is a promising cancer treatment target.

Pancreatic cancer stem cells (CSCs) are involved in promoting pancreatic cancer invasion and metastasis. CSCs are influenced by protease activation receptor 1 (PAR1) by inducing CSC-like properties in Aspc-1 cells. Therefore, doxycycline has been reported to inhibit PAR1, which effectively inhibits the CSC-like properties of pancreatic cancer cells and activation of the FAK/PI3K/AKT pathway, and enhances the therapeutic effect of 5 FU [33].

The role of protease-activated receptor 2 (PAR2) in gefitinib resistance was investigated, and its expression was found to be significantly increased when non-small-cell lung cancer (NSCLC) cells or tumour tissue exhibited gefitinib resistance. PAR2 was thus inhibited, suggesting a reversal effect in gefitinib resistance, in that gefitinib modulates EGFR transactivation, cell viability, migration, and apoptosis in gefitinib-sensitive and -resistant NSCLC cells. The study showed that the combination of gefitinib and PAR2 (P2pal-185) significantly blocked ERK phosphorylation and epithelial mesenchymal transition (EMT) compared to gefitinib alone. PAR2 was proposed as a novel target and pathway to overcome gefitinib resistance in NSCLC [34]. Signal Transducer and Activator of Transcription 3 (Stat 3) was introduced as a promising target for the treatment of breast cancer. The novel Stat 3 inhibitor, named Statmp-151, was investigated in the breast cancer cell lines MCF-7 and MDA-MB-231 and in the murine breast cancer cell line 4T1. The results showed that Statmp-151 could be a potential drug for the treatment of breast cancer [35].

The article "Heat Shock Protein 90 (HSP90) Inhibitors as Anticancer Medicines: A Review on the Computer-Aided Drug Discovery Approaches over the Past Five Years" was published in 2022. Journal: Comput Math Methods Med.

### 2.1. Overview of Heat Shock Protein

Heat shock proteins (HSPs) are a family of very abundant, essential, and evolutionarily conserved molecular chaperones. They maintain cellular homeostasis in response to stimuli that promote protein denaturation, such as hypoxia, anoxia, high temperatures, drugs, and other chemical compounds. HSP molecular mass, their subgroups, and cancer development are summarized in Table 1.

HSPs are categorised according to their molecular mass, with HSP70 being a subgroup of HSPs with a molecular weight of 70 kDa. HSP27, HSP40, HSP60, HSP70, HSP90, and large HSF are the main groupings categorised on the basis of their molecular weight. There has been a significant need to identify these large, overlapping proteins, as the number of HSP members is increasing and their names are confusing, as they are likely to have a high degree of similarity in some situations but differ greatly in others. HSPs are thought to play a key role in the molecular pathways that contribute to the growth and spread of cancer. HSPs may also have clinical applications as biomarkers for cancer diagnosis and disease progression assessment or as therapeutic targets for cancer therapy.

HSPs could be used as therapeutic targets in the treatment of cancer, leading to the development of new chemotherapeutic agents. HSP70 and HSP90 are the two best-studied members of the HSP family. The proteins GRP78 (a member of the HSP70 family) and HSP90 are targeted by most of the new cancer drugs currently being developed. Some of these drugs have been tested in clinical trials and have been shown to be effective against cancer cells in vitro and in animal xenograft models in vivo. It is not yet clear why cancer cells require different amounts of HSPs than normal cells, and more knowledge could lead to the discovery of a therapeutic window for the development of more effective and less toxic HSP inhibitors against cancer. HSP inhibitors could cause serious organ-specific toxicity (liver or eye toxicity) that is difficult to treat. It may be possible to circumvent the organ-specific toxicities of HSP inhibitors by identifying HSP functions that are specific to cancer cells. Some HSP inhibitors may be ineffective against cancer. To control cellular processes, members of the HSP family communicate and coordinate in a signalling network. When one HSP is inhibited, other HSPs may be overexpressed to compensate for the inhibitory effect of the single HSP inhibitor. For example, inhibition of HSP90 leads to overexpression of HSP27 and other HSPs, resulting in a heat shock response. The nomenclature and classification of human HSPs can be further improved to support functional descriptions of HSPs and drug discovery.

The article "Heat Shock Protein 90 (HSP90) Inhibitors as Anticancer Medicines: A Review on the Computer-Aided Drug Discovery Approaches over the Past Five Years" was published in 2022. Journal: Comput Math Methods Med.

Tumours in which HSP90 is overexpressed include pancreatic, ovarian, breast, lung, and endometrial cancers, squamous cell carcinoma of the oropharynx, and multiple myeloma [36–38]. In lung cancer, oesophageal cancer, bladder cancer, melanoma, and leukaemia, high expression of HSP90 has been shown to be a predictor of poor prognosis [39, 40]. HSP90 is a potential therapeutic target to suppress tumour development and progression as it plays a critical role in cancer biology, and many HSP90 inhibitors have been explored in clinical trials. As anticancer drugs, HSP90 inhibitors offer several advantages because many signalling proteins are HSP90 client proteins, HSP90 inhibitors can act on numerous signalling pathways simultaneously. Therefore, anti-HSP90 therapy is less likely to lead to tumour cell survival than therapy with only one target protein.

HSP90 is the most abundant chaperone protein in eukaryotes, accounting for around 1% to 2% of cytosolic proteins [41]. Under a range of intracellular and extracellular stressful situations, HSP90 supports the proper folding of newly generated proteins and helps in refolding denatured proteins [42]. The heat shock proteins generally are molecular chaperones that play key roles in many aspects of life. They are involved in the refolding of misfolded proteins, which helps to maintain cellular homeostasis. Heat shock factor (HSF) is activated in response to environmental stress and binds to heat shock elements (HSEs), increasing HSP translation and consequently high levels of HSP synthesis [43]. The heat shock protein 90 (HSP90) molecular chaperone occurs ubiquitously in eukaryotes and prokaryotes, where it plays a significant role in the maintenance of cell stability [44, 45]. Reliant on ATP, HSP90 is involved in activation, proper folding, assembly, transportation, conformation preservation, and breakdown of target proteins [46, 47]. However, these target proteins encompass many elevated or transmuted carcinogenic proteins, including p53 and hTERT, some of which are associated with cancer characteristics [48, 49]. These customer proteins in tumour generation, growth, invasion, and metastasis make HSP90 an appealing therapeutic cancer target [50, 51]. The overexpression of HSP90 has been observed in patients with cancer, and it has been observed that HSP90 triggers the unstable harmful kinase functions, which enhance carcinogenesis [52, 53]. Thus, highly efficient inhibitors are developed and synthesised for the treatment of HSP90-associated cancers. Therefore, the chemical bonding of inhibitors to HSP90 leads to customer protein breakdown that causes improper protein folding, which blocks tumourigenesis and escapes the drawbacks of drug resistance [54]. In such an instance, the oncoprotein implicated in several carcinogenic pathways is concurrently eliminated, creating a combinative tumour attack and significantly increasing the cancer cure rate. HSP90 inhibitors, therefore, have positive applications in the treatment of tumours [43, 55].

The article "Heat Shock Protein 90 (HSP90) Inhibitors as Anticancer Medicines: A Review on the Computer-Aided Drug Discovery Approaches over the Past Five Years" was published in 2022. Journal: Comput Math Methods Med.

## 3. The Structural Description of HSP90

The HSP90 proteins exist as homodimers where an individual monomer comprises three domains: the N-terminal domain, middle domain, and C-terminal domain (Figure 1) [56]. The N-terminal domain, which is a member of the GHKL superfamily, constitutes the major ATPase domain of HSP90. The N-terminal domain possesses a super-charged linker part with varying size (length), having a similar structure with gyrase, topoisomerase, and histidine kinase. It also constitutes other isoforms and species that link it to the middle domain [56–59]. The middle domain performs a significant function in hydrolysing the adenosine triphosphate (ATP) [60]. The C-terminus is responsible for the formation of the significant dimer interface of the HSP90. The Met-Glu-Glu-Val-Asp (MEEVD) motif, a fundamental interaction site for a subset of cochaperones with tetratricopeptide repeat (TPR) domains, is also found at the C-terminus [61].

Biological research has shown that a polypeptide is a homodimer where each monomer consists of three conserved regions that are flexibly related (N-, M-, and C-terminal domains). The N-terminal domain includes the nucleotide (ATP and ADP) and drug binding cleft, generally known as the “Bergerat fold” that is shut by a molecular “cork” of amino acids upon ATP binding and opens when an adenosine diphosphate (ADP) is attached. The middle domain is resistant to proteolysis and is designed to bind ATP's client proteins, a few cochaperones, and *π*-phosphate [60]. HSP90's ATPase activity is unquantifiable when that specific protein segment is absent and the site of protein dimerization is the C-terminal domain where a pentapeptide motif (Met-Glu-Glu-Val-Asp or MEEVD) that serves as a tetratricopeptide repeat (TPR) acceptor containing cochaperones is found. At the atomic level, the arrangement of this region, whose abstraction does not significantly disturb the functionality of the HSP90 protein, has yet to be solved [64, 65].

## 4. Development of Heat Shock Protein 90 Inhibitors

The process responsible for protein regulation of the cells known as homeostasis or proteostasis helps in the constant adoption of the cells to dynamic environments. HSP90 as molecular chaperones help proteins adopt and fold while avoiding misfold and aggregates resulting from stress [56]. The activities of HSP90 as chaperones and cochaperones are complex due to the conformational dynamism. HSP90 modulations appear to be preferred due to the competitive inhibition of the targeted N-terminal adenosine triphosphate pocket [56, 66]. Hitherto, among the 19 N-terminal targeted HSP90 inhibitors that made it to the clinical trials, none has been approved by FDA. This is because of harmful health effects such as the heat shock response (HSR) induction [63].  Figure 2 shows 2D structures of some of the failed N-terminal HSP90 inhibitors at the clinical trials. Compounds known as “C-terminal inhibitors,” which exploit several ways to control HSP90 function, have been produced as alternatives, either as natural product-based counterparts or through rational design [56]. One method of manipulating molecular chaperones is to use inhibitors produced from novobiocin to target the HSP90 C-terminus. Novobiocin structure-activity relationships have led to the discovery of neuroprotective or cytotoxic chemicals. C-terminal inhibitors are the only ones that can distinguish a prosurvival heat shock response from a cytotoxic reaction caused by client protein degradation [66].

The article "Heat Shock Protein 90 (HSP90) Inhibitors as Anticancer Medicines: A Review on the Computer-Aided Drug Discovery Approaches over the Past Five Years" was published in 2022. Journal: Comput Math Methods Med.

Over the years, researchers explored the use of natural products in the development of HSP90 inhibitors. Delmotte and Delmotte-Plaquee discovered radicicol (RD) as an extract from monosporium border and used it as a macrocyclic lactone antibiotic [63, 67]. In 1998, Schulte et al. identified radicicol as a competitive HSP90 inhibitor to geldanamycin (GA) [68]. Radicicol adoption of folding (perpendicular instead of parallel) conformations using the macrocyclic and aromatic rings differentiates it from geldanamycin. However, it is like radicicol in mimicking the conformational interactions with aspartate 93 (Asp93). Nevertheless, *in vivo* studies revealed some loopholes in radicicol's anticancer potency due to its short half-life and fast metabolic reactions [63, 69]. Therefore, inhibiting HSP90 with GA has decreased cancerous cells' growth and the breakdown of oncogenic proteins [70]. Analysis of the crystal structure determined the binding site for GA and RD within HSP90 in the N-terminal ATP-binding domain and mimicked the open ADP-binding conformation [71]. While GA and RD effectively targeted and disturbed HSP90 activity, their toxicity, and low stability, their clinical application was unsuccessful.

### 4.1. HSP90 N-Terminal Inhibitors

GA and RD selectivity towards HSP90 is due to HSP90's special N-terminal ATP-binding Bergerat fold geometric pocket, contained in the GHKL subgroup of ATPases [72, 73]. Less toxic and highly stable inhibitors within the ATP-binding pocket emerged from this selectivity to mimic GA and RD interactions. The earliest small-molecule inhibitor of HSP90 to reach clinical trials was a chemical analogue of GA (Figure 3), 17-allamino-17-demethoxy geldanamycin (17-AAG). This compound substituted the moiety 17-methoxy with a group 17-alkylamino to reduce toxicity [74, 75]. Although anticancer efficiency was demonstrated in phase I clinical trials, particularly when combined with trastuzumab in HER-2–positive breast cancer patients, the development of 17-AAG was terminated because of poor aqueous solubility and patent problems [76, 77]. Other analogues of benzoquinone ansamycin used in clinical trials include 17-DMAG, IPI-504, and 17-AG, and their structures are shown in Figure 3. The IPI-504 analogue was the most promising as it proceeded to clinical trial phases II and III. IPI-504 is a reduced quinone variant of GA, showing heightened HSP90 sensitivity and decreasing liver toxicity in patients.

The article "Heat Shock Protein 90 (HSP90) Inhibitors as Anticancer Medicines: A Review on the Computer-Aided Drug Discovery Approaches over the Past Five Years" was published in 2022. Journal: Comput Math Methods Med.

Nonetheless, IPI-504 progress was halted due to ineffectiveness in clinical trials [77]. There are no benzoquinone ansamycin compounds left on clinical review. Radicicol imitates HSP90's ADP-bound configuration and interacts similarly with Asp93 geldanamycin. Contrastingly, RD is oriented differently to GA when binding and has a higher degree of binding to the ATP pocket [71, 78]. Although not as structurally remarkable as GA, RD also takes on a folded configuration, with an essentially perpendicular rather than parallel macrocycle and aromatic ring [78]. However, RD does not exhibit antitumour activity because of its rapid in vivo metabolism [69]. Several synthetic analogues were produced by employing established conformational determinants of the RD-HSP90 bond complex. This resulted in the development of KF25706, a stable metabolic compound that demonstrated antiproliferative effectiveness in numerous human cancer cell lines and xenograft rodent models [79]. Although ideal for application, the complex nature of KF25706 has rendered it challenging for upscaling development. In addition to being vital for the inhibition of HSP90, the behaviour of RD's resorcinol moiety appears to be analogous to that of ATP's adenine ring. Several inhibitors have targeted this pharmacophore using the resorcinol ring and are undergoing clinical evaluation. It has been shown that STA-9090 (ganetespib), developed by Synta Pharmaceuticals Corp., is a resorcinol triazole molecule that has a high degree of binding with HSP90 and incapacitates it at as low concentrations as 0.01 *μ*M.

The article "Heat Shock Protein 90 (HSP90) Inhibitors as Anticancer Medicines: A Review on the Computer-Aided Drug Discovery Approaches over the Past Five Years" was published in 2022. Journal: Comput Math Methods Med.

Moreover, STA-9090 shows augmented invasion of tumours with low toxicity [79]. Rowlands et al. assessed a collection of 56 000 compounds and identified CCT018159, a molecule that includes the resorcinol-anchoring unit of radicicol [80–82]. Additional development of CCT018159 contributed to the formation of NVP, a resorcinol isoxazole amide approved by Novartis for clinical evaluation. More analogues of resorcinol include KW-2478 (Kyowa Hakko Kirin Pharma) and AT13387 (Astex). While analogues of benzoquinone ansamycin and radicicol are yet to be licensed for clinical application, the binding pocket reactions uncovered were utilised, and those compounds have been beneficial to developing an extra category of HSP90 inhibitors. The first fully synthetic derivatives produced were the purine-based compounds. These compounds utilised the folded conformation that GA and RD adopted following attachment to HSP90. Further studies of fully synthetic derivatives and their interactions with HSP90 contributed to PUH71 synthesis. This compound is affinitive of oncogenic cells and is only required to inhibit HSP90 activity at low concentrations. PU-H71 is currently under review for patients with advanced malignancies in a phase I clinical trial [83–85].

### 4.2. HSP90 C-Terminal Inhibitors

A second ATP-binding pocket was discovered inside the C-terminus of HSP90 using nucleotide affinity cleavage. The primary discovered C-terminal inhibitor was the natural product novobiocin [86, 87]. The novobiocin interaction site is close to the domain of C-terminal dimerisation and binds in a curved position, synonymous with ADP. Novobiocin's interaction with the C-terminus led to target protein breakdown, while its interaction with HSP90 remains unsteady [88]. The novobiocin structure was used to synthesise compound A4 and its analogues. These A4 analogues were coumarin-modified ring systems that mimic adenine and guanine with additional strategically positioned hydrogen bond acceptors and donors to suit higher specificity into the pocket [89]. The most potent novobiocin analogue produced was KU-174, designed to imitate the ATP-bound conformation [90]. This compound has demonstrated potency in several cancer cell lines as it breaks down clients without heat shock response (HSR) [91]. The platinum-comprising chemotherapeutical cisplatin and the microtubule stabiliser taxol are other C-terminal inhibitors [92]. Presently, there is no FDA-approved C-terminal HSP90 inhibitor, which appears to be of much concern to the pharmaceutical industries and scientists. There is, therefore, the need for more resources to be channelled towards this area of research. Interestingly, one of the challenges of N-domain-targeted agents is addressed by the ability of these compounds to inhibit HSP90 function without HSR induction, making C-terminal inhibitors compounds of interest for future investigation and exploration.

The article "Heat Shock Protein 90 (HSP90) Inhibitors as Anticancer Medicines: A Review on the Computer-Aided Drug Discovery Approaches over the Past Five Years" was published in 2022. Journal: Comput Math Methods Med.

### 4.3. Middle Domain Inhibitors

Sansalvamide A (San A) is an isolated cyclic pentapeptide from the sea fungus Fusarium species [93]. Sansalvamide A attaches to the middomain N-terminal fragment of HSP90 and exerts the ability to allosterically interrupt the contacts of C-terminal binding cochaperones and client proteins [93]. Interestingly, Di-Sansalvamide A (Di-San A), a dimerised version of San A, was found to bind HSP90's C-middle domain, indicating that Di-San A physically averts C-terminal binding clients from being bound [93]. Three compounds derived from San A, H-10, H-15, and LY-15, have been investigated in melanoma cells as possible inhibitors of HSP90. Such agents inhibited concentration- and time-dependent melanoma cell line growth. In addition, LY-15 and H-10 induced apoptosis-related mitochondrial pathways associated with caspase-3 and caspase-9 activation but not caspase-8 [94–96].

### 4.4. Some HSP90 Inhibitors in Clinical Trials

While the compounds currently in clinical trials have a wide range of structures, a closer look reveals that they can generally be categorised based on their similarity to GA, RD, or the purine scaffold. Only SNX-5422 does not fall into any of these classifications (Figure 2). As is common in drug discovery, natural products play an important role in lead discovery. GA in the case of HSP90, the active compounds of SNX-5422, RD, and ATP have played an important role in the development of small-molecule HSP90 inhibitors. None of these agents are acceptable as a therapeutic, but they have all served as good lead molecules or starting points for the majority of drugs currently being tested in clinical trials (Table 2).

## 5. Molecular Reactivity, Allosteric Dynamics, and Allosteric Design

The HSP90 plays a significant role in numerous metabolic pathways associated with cancer. Numerous trials targeting HSP90 have been conducted in drug discovery departments. In addition, several HSP90 inhibitors have been discovered but failed due to toxicity issues. Therefore, researchers have introduced allosteric perturbation as an alternative strategy to pharmacologically induce HSP90 ATPase activities and closure dynamics while modulating tumour cell death [98–100]. Furthermore, several advanced computational methods have been used in combination with experimental approaches to offer atomistic insights into the mechanistics of allosteric ligand recognition and its *in vivo* and *in vitro* processes, starting from the fully unbound state of HSP90 [101–103]. Stetz et al. [103] used a combination of molecular simulations and other studies of reaction experiments to disrupt the HSP90 conformation with structural analyses and coefficients to characterize the practical function of posttranslational modification (PTM) focal sites. The findings revealed that in the HSP90 conformation, a limited number of conserved PTMs serve as global biological mediators of allosteric dynamics and conversation, while maximally flexible PTM sites act as companions and sensors of allosteric structural changes. In 2020, Stetz et al. [102] examined the mechanism of allosteric interaction between HSP90 and Cdc37 phosphorylation sites during cartridge splicing. To quantify the heterogeneous consequences of phosphorylated sites and kinase-precise conversion switches, researchers used a combination of evolutionary assays, crude molecular simulations with noise-based fully collaborative modeling, and analyses of unbound and determinate HSP90 and Cdc37 systems. The findings show that the kinase-precise phosphorylation switches that convey signals to HSP90 vary their regulatory characteristics in part in response to current atopic predisposition. To see the transmission molecules inside the form and in HSP90, Astl et al. [101] employed an integrated laptop version with evolution and coefficient assessment, experimental protein linkage and structure modelling, molecular simulation, strength evaluation, and community modeling.

The article "Heat Shock Protein 90 (HSP90) Inhibitors as Anticancer Medicines: A Review on the Computer-Aided Drug Discovery Approaches over the Past Five Years" was published in 2022. Journal: Comput Math Methods Med.

They devised a network chain mechanism to ensure uniform coherence between compliance switches and identified important regulatory checkpoints that facilitate interactions and long-term dialogues with chaperones. The findings of this research add reveal further insights of the allergic law of HSP90 chaperones, as well as a model for the basic mechanism of conversation and a version of HSP90 with binding partners in the practical cycle. The tight ATPase response inside the vibrant site is related to the global structural and conformational dynamics of HSP90, according to large-scale biophysical investigations and molecular simulations. These findings offer a mechanistic model for the coupling of protein dynamics and catalysis and in HSP90, as well as a test of how the effects of extended coupling can affect enzymatic activity.

Computational modelling and computer-aided drug design have immensely contributed to the successful development of drugs, especially in the contemporary pharmaceutical and drug industries [104]. Integrating computer-aided drug design (CADD) into the development of HSP90 has contributed to the enhancement of selective drug targeting with reduced toxic and off-target effects [1]. Computational methodologies contribute significantly to the study of biomolecular structures and function [105]. This is due to the vast number of therapeutic receptor X-ray structures existing in the present day. Conventionally, designing novel drugs is usually a cumbersome, costly, and prolonged process. However, CADD methods (Figure 4) have constructively enhanced multitasking processes involved in drug development such as homology modelling, analysing the interacting proteins, predicting the binding sites, developing and validating the pharmacophore, molecular docking, and molecular dynamic simulations [1]. Some of these CADD are briefly described below.

The article "Heat Shock Protein 90 (HSP90) Inhibitors as Anticancer Medicines: A Review on the Computer-Aided Drug Discovery Approaches over the Past Five Years" was published in 2022. Journal: Comput Math Methods Med.

### 5.1. Homology Modeling

Homology modelling has significantly been helpful in modelling undetermined structures of HSP90 enzymes. Nevertheless, some already determined experimental structures have been stored and saved in the Protein Data Bank (PDB) [106, 107]. Formerly, the investigation of interatomic and intermolecular properties of HSP90 was limited [63]. Recently, researchers have explored the molecular modelling method in designing three-dimensional models of HSP90, which have provided a substantial understanding of its structural and mechanical dynamic properties [108].

### 5.2. QSAR

Quantitative structure-activity relationship (QSAR) methods are applied to estimate the correlation between physicochemical parameters, structures of chemical compounds, and their biomolecular properties [109]. QSAR has successfully been used to design new and potent drugs in the pharmaceutical and drug industries. As a computer-aided drug design method, it has helped design potent HSP90 drugs and inhibitors [107, 110, 111].

### 5.3. Molecular Docking

This CADD technique has been employed in predicting and evaluating the ligand-receptor binding poses and modes with the receptor's acting sites. The process entails docking, subsequently scoring the various poses and applying them to determine and calculate binding free energies [112]. This docking technique has been pivotal in computational drug discovery and modelling, such as designing HSP90 selective inhibition [113, 114]. Molecular docking extends to methods used to decipher the binding mechanism of small receptor ligands (macromolecules) [105, 115]. It is typically executed on structure-based rational drug design to classify precise small-molecule ligand conformations and approximate the frequency of interactions between ligands and proteins [116, 117]. The Cartesian coordinates of different receptors and ligands are utilised throughout the docking process to predict an appropriate conformation of the ligands for the resultant complex of ligand and receptor. To measure the ligand-receptor binding energy, molecular mechanics is used. Ligands and corresponding receptors interact dynamically, based on the molecular lock and critical method [118, 119]. The binding energies of the different ligands and receptors are compared to the inhibitor's bioactivity against the particular enzyme [120].

The article "Heat Shock Protein 90 (HSP90) Inhibitors as Anticancer Medicines: A Review on the Computer-Aided Drug Discovery Approaches over the Past Five Years" was published in 2022. Journal: Comput Math Methods Med.

### 5.4. Virtual Screening

Virtual screening involves the utilisation of the CADD in obtaining active lead molecules (compounds) from a considerable deposit or library of compounds. The method entails analysing three-dimensional structures of compounds resulting experimentally via X-ray crystallography or nuclear magnetic resonance (NMR) [112]. Virtual screening has been applied in the design of new HSP90 drugs with high selective inhibition [121].

### 5.5. Pharmacophore Development and Validation

Pharmacophore modelling has been used in the design of lead compounds when the structural properties of the protein are not resolved [122]. This technique has been employed in the discovery of compounds with the desired and selective inhibition [122, 123]. This technique has been in the concept of CADD, virtual screening, and pharmacophore development which have lately been useful in drug repurposing. This approach has been helpful in the development of HSP90 inhibition towards cancer therapy [124].

### 5.6. Molecular Dynamic (MD) Simulation

This technique investigates the dynamic mechanisms of the ligand-protein complex under different environments and conditions [125]. Molecular dynamic simulation has been extensively valuable for understanding proteins and other biomolecular compounds with regard to structural conformations and therapeutic purposes [126]. They were employing the instruments of molecular dynamic simulations in the development of HSP90 inhibitors [126]. The MD simulation binding energy evaluation and other postanalyses have been employed to validate the efficacy and potency of the HSP90 inhibitor-receptor complex [127]. Hitherto, researchers have yet to extensively explore the promising potentials of employing the CADD in designing particular and selective covalent heat shock protein90 inhibitors [128, 129].

### 5.7. Computational Studies (2016-2021)

Computational modelling and the application of computer-aided drug design (CADD) methods have been widely utilised to discover highly specific inhibitors for HSP90 towards cancer therapy [130]. In 2016, Mahmoud et al. discovered new HSP90 inhibitors by extensively employing CADD techniques such as pharmacophore modeling, molecular docking, QSAR, and virtual cocrystallisation pharmacophore [131]. The study identified twenty-four hits that showed HSP90 inhibition potentials with fifteen others having lower IC50 in micromolar [131]. In another research in 2016 by Baby et al., the authors employed the combinatory techniques of pharmacophore development and molecular docking in the identification of antagonist compounds of HSP90. The identified HSP90 antagonist compounds were chosen from heterocyclic molecules utilising GOLD 3.1 [122, 132]. Two inhibitors, Q1G and T21 (Figures 5(a) and 5(b)), had strong binding affinities and inhibitory effects, according to the findings. Q1G produced a network of H-bonds with the amino acid residues Asp93, Ser52, and Tyr139, whereas T21 generated H-bond interactions with Tyr139 and Asp93, indicating that these are important residues for HSP90 inhibition [122, 132]. Two hydrogen bond donors, two hydrogen bond acceptors, and two hydrophobic characteristics made up the best pharmacophore model [122, 132]. Furthermore, the molecular processes of HSP90 allosteric activation were discovered using MD simulations in conformational research by Vettoretti et al. This research also highlighted the structural consequences of allosteric modulation on HSP90, as well as its dynamical features in the active state, offering useful information for the development of new functional modulators [133].

The article "Heat Shock Protein 90 (HSP90) Inhibitors as Anticancer Medicines: A Review on the Computer-Aided Drug Discovery Approaches over the Past Five Years" was published in 2022. Journal: Comput Math Methods Med.

In 2017, Abbasi et al. predicted novel HSP90 inhibitors from 3,4-isoxazolediamide scaffold through combined computational techniques of quantitative structure-activity relationship, molecular docking, and subsequent MD simulations [134]. The importance of size, shape, symmetry, and branching of HSP90 inhibitory molecules was evident from the results. Docking studies showed that 2 hydroxyl groups in the resorcinol ring were important and necessary for the complex affinity. The orientation of the three groups was associated with the substitution of different R groups. The molecular dynamic (MD) simulation results were a comparison of a new compound and a best synthesised compound, where the novel compound (Figures 5(c)–5(e)) settled in an active site with lower binding energy than the best synthesised. Similarly, Garg et al. validated the effectiveness of the structure-activity relationship (SAR) method in the development of new C-terminal HSP90 inhibitors. The biological properties of these novel HSP90 inhibitors were further evaluated [130]. Again in 2017, Kumar et al. applied virtual screening of a library of compounds in the identification of potent molecules that could inhibit the oncogenic HSP90 interactome connected with breast cancer. This investigation identified 5 active lead compounds with appreciable binding energies in the range of -8.7 kcal/mol^−1^ to 10.7 kcal/mol^−1^ [104].

The article "Heat Shock Protein 90 (HSP90) Inhibitors as Anticancer Medicines: A Review on the Computer-Aided Drug Discovery Approaches over the Past Five Years" was published in 2022. Journal: Comput Math Methods Med.

In 2018, Terracciano et al. came up with the discovery of two novel potent C-terminal HSP90 inhibitors [135]. The two novel molecular species induced the death of cancerous cells while significantly downregulating HSP90. These new HSP90 inhibitors displayed a high capacity for interfering with the region of the HSP90 C terminal, which resulted due to the poor success of traditional N-terminal domain inhibitors, and an alternate inhibitory method was provided [135–139]. These discoveries were attained by employing exceptional refinement, molecular docking, and subsequent molecular dynamic simulations [135].

Sepehri and Ghavami studied tetrahydropyrido[4,3-d]pyrimidine derivatives (Figure 5(f)) as HSP90 inhibitors through molecular docking and 3D-QSAR CoMFA [140]. According to extracted contour maps or the CoMFA model, three inhibitors were obtained and docked to the N-terminal domain binding site of the HSP90. These compounds acquired essential binding energies [140]. Furthermore, Abbasi et al. also in 2018 predicted new HSP90 inhibitors based on isoxazole scaffold (Figure 5(g)) through 3D-QSAR, molecular docking, and molecular dynamics [141]. Using comparative molecular field analysis (CoMFA) and comparative molecular similarity indices analysis (CoMSIA), the steric and electrostatic contour maps were made and hydrophobic and hydrogen bonds established, while donors and acceptors were generated. Consequently, novel compounds were predicted. The predicted compound binding modes in the HSP90 binding site were investigated and evaluated using molecular docking and molecular dynamics (MD), which were found to be stable in the binding site [141].

In 2019, Mettu et al. designed and synthesised novel pyrazolyl 2-aminopyrimidine derivatives (Figure 5(h)) as HSP90 inhibitors, which were evaluated using molecular docking studies [142]. The studies showed that synthesised molecules retained all the essential binding interactions with HSP90 [142]. In another study in 2019, Rampogu et al. focused on natural compounds as possible inhibitors of HSP90 for breast cancer-pharmacophore-guided molecular modeling [143]. The database of 3210 natural phytochemicals was assessed to retrieve the potential inhibitors after thorough confirmation of the model pharmacophore. Sequel to the screening, 135 phytochemical compounds were retrieved and further sorted by drug-likeness factors, including Lipinski's role of five, ADMET properties, and molecular docking-based scoring [144, 145]. Three phytochemical molecules obtained from docking studies displayed better properties than investigated clinical therapeutics. In addition, the hit compound and reference compounds with docking scores of 48.27 (geldanamycin), 40.90 (radicicol), 73.04 (Hit1), 72.92 (Hit2), and 68.12 (Hit3) (Figures 5(i) and 5(j)) were validated for their binding stability through molecular dynamics [143].

The article "Heat Shock Protein 90 (HSP90) Inhibitors as Anticancer Medicines: A Review on the Computer-Aided Drug Discovery Approaches over the Past Five Years" was published in 2022. Journal: Comput Math Methods Med.

In 2020, Nazar et al. applied an in silico approach, molecular docking, molecular dynamic simulations, and binding free energy calculations to understand HSP90 inhibition mechanisms to identify novel cancer therapeutics [125]. On the grounds of GOLD fitness score and orientation to docked HSP90 inhibitors with their analogues, they were designated as the superlative molecules. The interactions of these inhibitors with the HSP90 active site were observed to be significant. Molecular dynamics (MD) of top-docked molecules (Figures 5(k) and 5(l)) ensured a strong binding interaction between inhibition and the HSP90 active site. The results yielded new perceptions into the design of cancer-targeting HSP90 [125]. In another report, Nazar et al. designed new heat shock protein (HSP90) inhibitors by pharmacophore modeling and a virtual screening workflow was utilised to determine the molecule's key structure (ZINC02819805) (Figure 5(m)) [125]. Pyrazolopyranopyrimidine derivatives were designed through the optimisation of compound ZINC02819805. The key critical interactions between one of the designed compounds and HSP90 were deliberated by molecular dynamic simulation and displayed stability [125].

He et al. (2020) conducted in silico studies to design new vibsanin B derivatives (Figures 5(n) and 5(o)) and HSP90 inhibitors based on 3D-QSAR, molecular docking, and molecular dynamic simulation [146]. The directive information for structural information of the inhibitors was conducted from CoMFA and CoMSIA [147]. The stability of inhibitors in the binding site was evaluated through molecular docking and dynamics, which also suggested that numerous key residues had a significant contribution to the activity. The majority of virtually designed compounds in this research presented a sensible ADMET profile, which offered theoretical support for the structural medication of HSP90 [147, 148]. Godoy-Castillo et al. identified the naphthoquinone derivative inhibitor's binding site in HSP90 through an induced-fit docking, molecular dynamics, and 3D-QSAR study [149]. Molecular docking and dynamic simulations brought an understanding of the binding modes and the respective protein-inhibitor interactions. The results provided grounds for rational modifications of novel molecules founded from the quinone scaffold (Figure 5(p)), to create HSP90 inhibitors of high potency for high antitumour activity [149].

The article "Heat Shock Protein 90 (HSP90) Inhibitors as Anticancer Medicines: A Review on the Computer-Aided Drug Discovery Approaches over the Past Five Years" was published in 2022. Journal: Comput Math Methods Med.

Tomašič et al. also discovered new HSP90 C-terminal inhibitors using 3D-pharmacophore obtained from molecular dynamic simulations [150]. A suitable binding site was identified by pharmacophore models and virtual screening derived from a unique approach that allows one to derive and analyse ligand-protein interaction from molecular dynamic trajectories. Among the retrieved compounds from virtual screening, two compounds were biologically tested. A compound that offered a unique scaffold with promising properties for future synthetic optimisation and molecule development is required to evaluate HSP90 C-terminal domain as the focus of interest to develop anticancer drugs [151]. Shadrack et al. conducted a computational study on the role of water and conformational fluctuations in HSP90 in response to inhibitors [152]. The authors suggested docking practices for the repurposing of FDA-approved HSP90 drugs. The apo, holo, and receptor ensemble (relaxed complex) structures, the role of water, and HSP90 conformational modifications were described [152, 153]. Docking energies to the inclusion of water were reported to be more sensitive when executed on the crystal structure as contrasted with the RCS ensemble. The results serve as a possible basis for the development of HSP90 inhibitors [154]. Bekker et al. used a multicanonical molecular dynamic-based dynamic docking to thoroughly investigate the configurational space of an inhibitor binding to the N-terminal domain of HSP90 [155]. The dynamic docking method in this study effectively predicted the inherent binding site while thoroughly testing a wide configurational space, exerting an altering influence on the protein structure upon binding [155].

Cai et al. synthesised new pyrazole-containing imide derivatives (Figure 5(q)) and assessed them using molecular dynamic simulation [156]. The HSP90 was suggested as the probable drug target of these compounds with the assistance of pharmacophore and molecular docking. The stability of these compounds was evaluated by molecular dynamics [156]. Magwenyane et al. studied the structural and molecular insight into the remedial properties of radicicol (RD) and NVP-YUA922 (NVP) (Figure 6) by inhibition of cancer using DFT, molecular docking, and MD to understand the HSP90 N-terminal dynamics [63]. Density functional theory (DFT) calculations predicted NVP to have high favourability with solvation free energy at -23.3 kcal/mol and the highest stability energy of 75.5 kcal/mol for a major atomic delocalisation. Molecular dynamic (MD) assessment revealed high stability of NVP bound to HSP90 (NT-NVP) when compared to RD (NT-RD). The HSP90 protein displayed a greater binding affinity for NT-NVP compared to NT-RD, where the vital residues prominent in the binding are Gly 97, Asp 93, and Thr 184. The discoveries therein serve as constructive perceptions into HSP90 dynamics and will assist in the construction of potent new inhibitors for cancer therapy [63]. Dike et al. applied the in silico approach to identify small-molecule modulators to disrupt the HSP90-Cdc37 protein-protein interaction boundary for cancer therapy [157]. Four molecules were discovered from a collection of above 60 000 compounds. The molecular dynamic (MD) simulation elucidated that all four molecules were kept inside the interface and strong affection for HSP90-Cdc37. Therefore, the molecule in suggestion could be critical to successfully inhibit the HSP90-Cdc37 interface [157].

The article "Heat Shock Protein 90 (HSP90) Inhibitors as Anticancer Medicines: A Review on the Computer-Aided Drug Discovery Approaches over the Past Five Years" was published in 2022. Journal: Comput Math Methods Med.

In 2021, Mak et al. discovered two drug-like novel HSP90 CTD inhibitors by using virtual screening and intrinsic protein fluorescence quenching binding assays, preparing for future developments of novel therapeutics that utilise molecular chaperone inhibitors [151]. In another study, Rezvani et al. identified two new HSP90 inhibitors through the in silico techniques of molecular docking, MD simulations, and density functional theory [1]. Zinc15 structural queries were used to locate related compounds in HSP90 inhibitors in various clinical trials stages (78 percent). Twenty-nine small molecules were obtained and docked into an ensemble of HSP90-NTDs using a predetermined similarity cut-off. H-bond, hydrophobic, and salt bridge interactions were found to be determining forces in complex formation using molecular docking and intermolecular binding studies. The binding pocket of HSP90 was efficiently accommodated by compounds 19 and 20 due to their somewhat diverse conformations. Asn51 and Phe138 were discovered to be important residues that interacted with 19 and 20 in a stable manner [1].

Wang et al. employed the quantitative structure-activity relationship (QSAR) technique to investigate aminopyrazole-substituted resorcylate compounds as HSP90 inhibitors [158]. The new HSP90 inhibitors, aminopyrazole-substituted resorcylate compounds, have a wide range of HSP90 inhibitory action and were created to develop new antibacterial medications. The fungal selectivity of novel HSP90 inhibitors was predicted using a quantitative structure-activity relationship technique. The best linear model's *R* correlation coefficient was 0.89 and 0.11 and resulted in the development of two nonlinear models [158]. In another study, Tomašič et al. applied the three-dimensional pharmacophore profiling on selective DNA gyrase and HSP90 inhibitors [159]. The authors designed selective three-dimensional pharmacophore systems for GyrB, human topoisomerase II*α* (TopoII), and the HSP90 N-terminal domain (NTD) used as starting points for hit expansion and lead optimisation. Using their off-target pharmacophore modeling, they were able to predict the selective on-target binding of GyrB inhibitors. In vitro studies on HSP90 and TopoII for selected compounds 1 and 2 corroborated these findings. In vitro studies against E. coli DNA gyrase and human TopoII validated the prediction of selective HSP90 NTD inhibition for 3 and 4, which was also confirmed in in vitro assays against E. coli DNA gyrase and human TopoII. It was confirmed that designing three-dimensional chemical parameter-based pharmacophore models are useful instruments for predicting the activity and selectivity of known and novel HSP90 and GyrB inhibitors [159].

The article "Heat Shock Protein 90 (HSP90) Inhibitors as Anticancer Medicines: A Review on the Computer-Aided Drug Discovery Approaches over the Past Five Years" was published in 2022. Journal: Comput Math Methods Med.

Rezvan et al. used a Zinc15 structural interrogation to reveal comparable compounds (≥78%) in HSP90 inhibitors that were at different stages of clinical trials. Small molecules were found docked to an ensemble of HSP90 NTDs using a predetermined similarity cut-off. Two molecules with very different conformations were shown to be well tolerated in the binding pocket of HSP90. Asn51 and Phe138 were found to be important residues that interacted stably with compounds. Even though the basic mechanism of action of the proposed compounds is unknown and remains to be investigated, the results of this work point to critical structural features for future structure-guided optimisation towards potent inhibitors of HSP90-NTD [1].

## 6. Conclusion

There has been a paradigm change in recent years toward the development of highly selective inhibitors of oncogenic HSP90. This was important to overcome roadblocks that hampered the postclinical approval of already available medications, notwithstanding their efficacy in a variety of preclinical and clinical investigations. Conventionally, designing novel drugs is usually a cumbersome, costly, and prolonged process. However, CADD methods have constructively enhanced multitasking processes involved in drug development such as homology modelling, analysing the interacting proteins, predicting the binding sites, developing and validating the pharmacophore, molecular docking, and molecular dynamic. The application of modern CADD techniques to HSP90 research has yielded structural and molecular insights that have aided in the identification and improvement of new HSP90 inhibitors with increased selectivity and activity. Despite the progress made thus far, a new dynamic in silico techniques with experimental validations is still needed to get highly selective results. We also suggest an extensive investigation of advanced computational modelling of the three different domains of HSP90 for potent, effective inhibitor design with minimal off-target effects.

The article "Heat Shock Protein 90 (HSP90) Inhibitors as Anticancer Medicines: A Review on the Computer-Aided Drug Discovery Approaches over the Past Five Years" was published in 2022. Journal: Comput Math Methods Med.

## Figures and Tables

**Figure 1:** Diagram representing the three domains of HSP90 protein (crystal structure of HSP90 dimer with PDB ID: 2CG9 while the red dashed cycle highlights an ATP-binding pocket) as adopted from open-source journals [62, 63].

**Figure 2:** 2D structures of some of the failed N-terminal HSP90 inhibitors at the clinical trials.

**Figure 3:** 2D structure of HSP90 natural inhibitor, geldanamycin (GA), and derivatives.

**Figure 4:** Computational modeling and drug design methods employed for HSP90.

**Figure 5:** 2D structures of HSP90 inhibitors obtained and analysed via computational studies.

**Figure 6:** 2D structures of C-terminal and M-domain HSP90 inhibitors.

**Table 1:** The overview of heat shock proteins (HSPs) in cancer development.

Family	Cancer development
HSP27	Response to heat shock and recovery of damaged proteins, regulation of cytoskeleton dynamics Modulation of tumour initiation, progression, cancer stem cell programming, and metathesis by Hippo pathway Regulation of cancer development, EMT, cell proliferation, migration, and invasion Relation of poor prognosis and biomarker for cancer diagnosis

HSP40	Classified into DnaJB and DnaJC Regulation of protein folding, refolding, translation, translocation, and degradation Association with progression, growth, invasion, and metastasis in cancer DNAJ transcriptome analysis—relation of lymphatic invasion, infiltrative growth type, lymph node metastasis, cell proliferation, and progression in cancer

HSP60	Localization in mitochondria, relation of quality control (mitochondrial function, proteostasis, and transport and folding of mitochondrial proteins Function as a promoter and suppressor of cancer Regulation of cell growth, differentiation, invasion, metastasis, and mitochondrial biogenesis in cancer

HSP70	Five important family (HSP27, HSP70B, HSC70, Mortalin, and GRP78) Important roles in protein folding, homeostasis, and cell survival Association with cancer development, progression, malignancy, recurrence, and poor prognosis Regulation of cell proliferation, migration, invasion, apoptosis, and phenotype of cancer stem cells

HSP90	Relation to protein folding, stabilization, activation, and proteolytic degradation Modulation of tumour growth, adhesion, invasion, metastasis, angiogenesis, and apoptosis Association with cancer development, progression, and poor prognosis

HSF1	Master regulator of all heat shock responses Modulation invasion, migration, and EMT of cancer Regulation of tumour growth, overall survival, apoptosis, and metabolism in cancer Association with cancer development, progression, and poor prognosis

The article "Heat Shock Protein 90 (HSP90) Inhibitors as Anticancer Medicines: A Review on the Computer-Aided Drug Discovery Approaches over the Past Five Years" was published in 2022. Journal: Comput Math Methods Med.

**Table 2:** HSP90 inhibitors in clinical evaluation [97].

Inhibitor	Company	Class	Route	Phase
Tanespimycin (17-AAG, KOS-953)	Kosan Biosciences/Bristol Myers Squibb	GA	IV	III
Alvespimycin (17-DMAG)	Kosan Biosciences/Bristol Myers Squibb	GA	IV oral	I
Etaspimycin (IPI-504)	Infinity Pharmaceuticals	GA	IV	III
IPI-493	Infinity Pharmaceuticals	GA	Oral	I
CNF2024/BIIB 021	Biogen Idec	Purine	Oral	II
MPC-3100	Myriad Pharmaceuticals/Myrexis	Purine	Oral	I
Debio 0932 (CUDC-305)	Debiopharm	Purine-like	Oral	I
PU-H71	Samus Therapeutics	Purine	IV	I
Ganetespib (STA-9090)	Synta Pharmaceuticals	Resorcinol-triazole	IV	II
NVP-AUY922 (VER-52269)	Novartis	Resorcinol-isoxazole	IV	II
HSP990	Novartis	Not reported but claimed as a follow-up compound to NVP-AUY922	Oral	I
KW-2478	Kyowa Hakko Kirin Pharma	Resorcinol	IV	I
AT13387	Astex	Resorcinol	IV oral	I
SNX-5422	Serenex/Pfizer	Indazol-4-one	Oral	I
DS-2248	Daiichi Sankyo Inc.	Not reported	Oral	I
XL888	Exelixis	Not reported	Oral	I

## Data Availability

The generated data used to support the findings of this study are included in the article.
